# Decreased MiR-128-3p alleviates the progression of rheumatoid arthritis by up-regulating the expression of TNFAIP3

**DOI:** 10.1042/BSR20180540

**Published:** 2018-07-31

**Authors:** Zhongbin Xia, Fanru Meng, Ying Liu, Yuxuan Fang, Xia Wu, Chunwang Zhang, Dan Liu, Guoqing Li

**Affiliations:** 1 Department of Rheumatology, Clinical Medical College, Yangzhou University, Yangzhou 225000, China; 2 Postgraduate School, Dalian Medical University, Dalian 116000, China; 3 Department of Pathology, Clinical Medical College, Yangzhou University, Yangzhou 225000, China

**Keywords:** inflammation, MiR-128-3p, NF-κB, Rheumatoid arthritis, TNFAIP3

## Abstract

**Background:** Rheumatoid arthritis (RA) is a inflammatory disease that characterized with the destruction of synovial joint, which could induce disability. Inflammatory response mediated the RA. It has been reported that MiR-128-3p is significantly increased in RA, while the potential role was still unclear.

**Methods:** T cells in peripheral blood mononuclear cell (PBMC) were isolated from the peripheral blood from people of RA and normal person were used. Real-time PCR was performed to detect the expression of MiR-128-3p, while the protein expression of tumor necrosis factor-α-induced protein 3 (TNFAIP3) was determined using Western blot. The levels of IL-6 and IL-17 were measured using enzyme-linked immunosorbent assay (ELISA). The expression of CD69 and CD25 was detected using flow cytometry. The RA mouse model was constructed for verification of the role of MiR-128-3p.

**Results:** The expression of MiR-128-3p was significantly increased, while TNFAIP3 was decreased, the levels of IL-6 and IL-17 were also increased in the T cells of RA patients. Down-regulated MiR-128-3p significantly suppressed the expression of p-IkBα and CD69, and CD25in T cells. MiR-128-3p targets TNFAIP3 to regulate its expression. MiR-128-3p knockdown significantly suppressed the activity of nuclear factor κB (NF-κB) and T cells by up-regulating TNFAIP3, while cells co-transfected with si-TNFAIP3 abolished the effects of MiR-128-3p knockdown. The *in vivo* experiments verified the potential role of MiR-128-3p on RA.

**Conclusion:** Down-regulated MiR-128-3p significantly suppressed the inflammation response of RA through suppressing the activity of NF-κB pathway, which was mediated by TNFAIP3.

## Introduction

Rheumatoid arthritis (RA) is a inflammatory disease that characterized with the destruction of synovial joints, which severely threatens human joint. It has reported that the progressed RA could further lead to disability. Even though great progression has been made on effective medications for RA, the disability rate that induced by RA was still high. Genetic studies have reported that the rheumatoid factors and several inflammatory cytokines played an important role in the mechanism of RA, while the etiology of RA remains unclear.

Immunity role of T cells plays a critical role in RA. The abnormally T cells often evoke the dysregulated expression of several inflammatory mediators, such as tumor necrosis factor-α (TNF-α), interleukin-1(IL-1), IL-6, and IL-17. The nuclear factor κB (NF-κB), a transcription factor, is involved in the inflammatory process of RA, and the NF-κB signaling pathway has been reported to conduct the inflammatory mediators of RA [1,2]. To interference, the activity of NF-κB signaling pathway could effectively protect body against the aggression of inflammation [3]. Therefore, to explore the potential role of NF-κB signaling pathway is important for further RA study.

Tumor necrosis factor-α-induced protein 3 (TNFAIP3), also known as A20, is a cytoplasmic zinc finger protein that was originally identified as a dual inhibitor of NF-κB activation. Mounting studies have reported that the TNFAIP3 played an important role in the inflammation [4–6]. A recent study demonstrated that the expression of TNFAIP3 was significantly decreased in RA, and regulated the expression of several key cytokines of inflammatory process via negatively regulating the activity of NF-κB signaling pathway [7,8]. While the potential role of TNFAIP3 on RA was still undocumented.

MicroRNA (miRNA) is a class of noncoding RNA (ncRNA) with the length of ~22 nucleotides and regulates gene expression at the post-transcriptional level by binding the 3′-UTR of targeted genes. Recently, much miRNAs have been reported to mediate the cell apoptosis, signaling transduction, body metabolism, and immune response. Plenty miRNAs, such as miR-146a [9], miR-155 [10], miR-16 [11], miR-23b [12], miR-203 [13], miR-124a [14], miR-346 [15], and miR-223 [16], have been reported to mediated the synovial fibroblasts, peripheral blood mononuclear cells and T cells in RA, indicating the potential role of miRNA in RA. MiR-128-3p has been widely studied in various diseases, such as esophageal squamous-cell cancer [17], lung cancer [18], and kidney inflammation [19]. Mounting studies have reported that MiR-128-3p served as a tumor suppressor gene [18,20]. While the expression of miR-128 was significantly higher in RA patients than that in control [21]. However, whether miR-128 mediated the regulation mechanism of RA was still unclear.

In the present study, we first examined the inflammation-related cytokines; then we conducted *in vitro* experiments to identify the potential mechanism of RA; finally, the *in vivo* experiments were performed to verify our results. Our aims were to explore the potential role of MiR-128-3p on RA, and the potential mechanism of inflammatory response on RA. The present study will provide great help for further clinical therapy of RA.

## Materials and methods

### Patients

Twenty patients, who are diagnosed with RA in our hospital, were recruited in the present study. Another 20 healthy volunteers were acted as control. The study were approved by the ethic committee of Clinical Medical College, Yangzhou University. All patients were assigned the informed consent. Blood was collected after 12 h at the last medicine taking to minimize the effects of the drugs.

### Isolation of T cells

To isolate T cells, the peripheral blood mononuclear cells (PBMCs) were separated from the blood samples. The blood was mixed with 2% dextran solution (Sigma, Japan) and cultured for 30 min in the room temperature. The supernatants were collected and layered using a density gradient centrifuge to separate the mononuclear cells. T cells were purified using antihuman CD3-coated magnetic beads. The concentration of T cells was cultured in RPMI-1640 medium containing 10% fetal bovine serum (FBS) at 37°C in a humidified atmosphere.

### The activation of T cells and flow cytometry

T cells were cultured as described above and stimulated for 18 h with anti-CD3 and anti-CD28 antibodies or PMA/ionomycin to check respectively CD69 and CD25 expression. CD69-PE (BD Biosciences; 585/42BP) and CD25-PE (ImmunoStep, Salamanca, Spain; 585/42BP) expression were measured by fluorescence activated cell storing (FACS). The details were described in the article of Dong et al. [22].

### Real-time PCR

The total RNA was isolated from T cells using the RNA Isolation Kit (Sigma-Aldrich), according to the manufacturer’s instruction. RNA quality was determined using the agarose gel electorphesis, and the concentration was detected using a Nanodrop Spectrophotometer. The cDNA was reverse transcripted using a QuantiTect Reverse Transcription Kit (Qiagen), according to the instruction. The real-time PCR was performed using an ABI Prism 7500 Fast Real-Time PCR system (Applied Biosystems, U.S.A.). Each experiment was repeated for three independent times, and U6 served as internal control.

### Western blot

Cells were lysed using the RIPA Lysis buffer. The protein concentration was determined using micro bicinchoninic acid (BCA) method. The proteins were separated using 10% SDS-PAGE, and the equal amount of protein was transferred to PVDF membrane and incubated with the primary antibodies at 4°C for 24 h. Then the PVDF membrane was incubated with the second primary at room temperature for 1 h. β-Actin served as internal control. The ECL chemiluminescence was used to visualize the protein bands.

### Luciferase reporter assay

The miRNA target interactions were based on the principle of the references [23,24]. The online TargetScan (v7.0; targetscan.org) was used to predict the potential binding site between MiR-128-3p and TNFAIP3 as described in the previous study [25]. To further identify the potential relationship, luciferase reporter assay was conducted. TNFAIP3 containing a wild-type or mutant 3′-UTR was constructed. HEK 293T cells were planted in 24-well plates, and the wild-type or mutant of TNFAIP3 and MiR-128-3p was co-transfected using Lipofectamine 2000. The activity was measured after 24 h using a Dual-Luciferase® Reporter Assay System (Promega Corporation, U.S.A.).

### Cell transfection

Cells were planted in a 24-well plate for 24 h, the inhibitor, mimic, and their negative control (synthesized in Invitrogen, Shanghai, China) were transfected to the cells using Lipofectamine 2000 (Invitrogen), and the concentration of MiR-128-3p inhibitor and mimic was 100 nmol/l.

### Enzyme-linked immunosorbent assay (ELISA)

The levels of IL-6 and IL-17 in the serum were detected using ELISA kit (USCN Life Science Inc., Wuhan, China). The samples were incubated with the enzyme-labeled antibody for 30 min at 37°C. The sulfuric acid of 2 M (0.05 ml) was used to suspend the reaction. The ultraviolet spectrophotometer (Eppendorf BioSpectrometer) was used to visualize the values with the OD = 450 nm.

### Animals

The C57BL/6 mice were purchased from the Experimental Animals center of Shanghai. The mice were aged at 4–6 weeks and weighted 20–30 g. The mice were cultured in a cozy environment and supplied with plenty of food and water. A 12 h day–night circle was also provided. The animal experiments were approved by Clinical Medical College, Yangzhou University.

### Establishment of RA mouse model

To establish the RA mice model, the mice were injected intradermally using 0.1 ml of an emulsion containing 100 μg of bovine type II collagen and complete Freund’s adjuvant (Arthrogen-CIA; Chondrex, Seattle, WA) into the base of the mice tail. After 2 weeks, 100 μg of type II collagen, dissolved and emulsified 1:1 with incomplete Freund’s adjuvant (Difco, Detroit, MI), was administered to the hind leg. To further identify the role of MiR-128-3p on RA *in vivo*, the RA mode was divided into two groups (*n*=6 in each group): negative control and miR-128 inhibitor group. MiR-128 inhibitor (60 nmol/l) was intravenous injection twice a week for 4 weeks.

### The arthritis score calculation

The RA score of hind feet of the rats was calculated to assess the inflammation level of arthritis. The details were as follows: 0 score, no arthritis symptom in hind feet; 1 score, red with soft tissue swelling was observed in one or two hind feet; 2 scores, red with soft tissue swelling was observed in three to four joints in hind feet; 3 scores, red with soft tissue swelling was observed in five or even more joints in hind feet; 4 scores, hind feet showed severe arthritis symptoms.

### Statistical analysis

All data were presented as means ± SD. Statistical differences were analyzed using student’s *t*-test for paired samples and ANOVA for multigroup samples. *P*<0.05 considered as statistical analysis.

## Results

### The expression pattern of MiR-128-3p and TNFAIP3 in clinical tissues

To learn the expression of MiR-128-3p and TNFAIP3 and the level of inflammatory cytokines in RA, the PBMCs of clinical RA patients were collected and the T cells were isolated. As is presented in Figure 1, the expression of MiR-128-3p was significantly increased (Figure 1A), while TNFAIP3 was decreased in T cells of RA patients compared with control (Figure 1B). In addition, the cytokines of IL-6 and IL-17 were markedly higher in RA patients rather than in control (Figure 1C). The results indicated that MiR-128-3p was higher in RA patients along with the inflammatory response. In addition, we analyzed the correlation between miR-128-3p expression and the clinical characteristics of RA patients. As presented in Table 1, the miR-128 expression was correlated with rheumatoid factor (RF), erythrocyte sedimentation rate (ESR), C-reactive protein (CRP), and mean disease activity score in 28 joints (DAS28), but did not correlated with age, sex, and disease duration.

**Figure 1:** The expression pattern of MiR-128-3p and TNFAIP3 in clinical T cells of RA (**A**) The expression of MiR-128-3p was determined using real-time PCR. (**B**) The expression of TNFAIP3 was measured using Western blot. (**C**) The levels of IL-6 and IL-17 were detected using ELISA; *P<0.05 vs. HC.

**Table 1:** Characteristics of RA samples

Demographics	Active RA (*n*=20)	Healthy (*n*=20)
Age (years), mean (range)	53 (26–77)	49.1 (21–78)
Sex, female/male	18/2	17/3
Disease duration (years), mean (range)	11 (2–23)	–
RF, positive/negative	15/5*	–
ESR (mm/h), mean (range)	65.23 (28–112)*	7.5 (6–17)
CRP (mg/l), mean (range)	69.62 (31–148)*	2.8 (1–8)
Mean DAS28	5.91 (4.3–7.1)*	–

Abbreviations: RF, rheumatoid factor; ESR, erythrocyte sedimentation rate; CRP, C-reactive protein; DAS28, disease activity score in 28 joints;

* *P*<0.05 represented the relationship between miR-128 expression and the clinical characters.

### MiR-128-3p knockdown significantly suppressed the signaling of NF-κB and decreased the activation of T cells

To explore the effects of MiR-128-3p on the pathway of NF-κB and the activation of T cells, the T cells were first activated and then transfected with MiR-128-3p inhibitor. The results presented that the expression of MiR-128-3p was significantly decreased (Figure 2A). MiR-128-3p knockdown significantly decreased the expression of p-IkBα, but did not affect the expression of IkBα (Figure 2B). Additionally, the MiR-128-3p inhibitor also suppressed the ratio of CD69 and CD25 (Figure 2C). Taken together, down-regulated MiR-128-3p suppressed the inflammatory response as well as the activity of NF-κB.

**Figure 2:** Effects of MiR-128-3p on the activity of NF-kB and T cells The activated T cells were transfected with MiR-128-3p inhibitor. (**A**) Real-time PCR was performed to determine the expression of MiR-128-3p. (**B**) Western blot was carried out to determine the protein expression of p-IkBα and IkBα. (**C**) The expression of CD69 and CD25 was measured using flow cytometry; *P<0.05 vs. NC.

### The relationship between MiR-128-3p and TNFAIP3

Online TargetScan predicted that MiR-128-3p could bind with the 3′-UTR of TNFAIP3 (weighted context++ score: −0.10; total context++ score: −0.11; aggregate PCT: <0.1). The luciferase reporter assay revealed that MiR-128-3p mimic significantly decreased the relative luciferase activity in WT-TNFAIP3 3′-UTR, while MiR-128-3p inhibitor dramatically promoted the relative luciferase activity in WT-TNFAIP3 3′-UTR (Figure 3B). Furthermore, MiR-128-3p mimic significantly decreased the expression of TNFAIP3, while MiR-128-3p inhibitor significantly promoted the expression of TNFAIP3, indicating that MiR-128-3p directly regulated the expression TNFAIP3.

**Figure 3:** The relationship between MiR-128-3p and TNFAIP3 (**A**) Online TargetScan predicted that MiR-128-3p bound with the 3′-UTR of TNFAIP3. (**B**) Luciferase reporter assay was performed to determine the role of MiR-128-3p on the luciferase activity. (**C**) Western blot was performed to determine the role of MiR-128-3p on TNFAIP3; *P<0.05 vs. pre-NC or NC.

### MiR-128-3p knockdown decreased the activation of NF-κB via up-regulating the expression of TNFAIP3

The activated T cells transfected with MiR-128-3p inhibitor significantly promoted the expression of TNFAIP3, while then co-transfected with si-TNFAIP3 abolished the effects of MiR-128-3p inhibitor (Figure 4A). T cells transfected with MiR-128-3p inhibitor decreased the expression of p-IkBα, while co-transfected with si-TNFAIP3 reversed the effects of MiR-128-3p inhibitor (Figure 4B). In addition, the MiR-128-3p inhibitor also decreased the cytokines of IL-6 and IL-17, while cells co-transfected with si-TNFAIP3 significantly reversed them (Figure 4C). Taken together, down-regulated MiR-128-3p promoted the expression of TNFAIP3, which further decreased the activation of NF-κB.

**Figure 4:** The role of MiR-128-3p knockdown on the activity of NF-κB (**A**) The expression of TNFAIP3 was determined using Western blot. (**B**) The expression of p-IkBα and IkBα was measured using Western blot. (**C**) The levels of IL-6 and IL-17 were determined using ELISA; *P<0.05 vs. NC; ^#^*P*<0.05 vs. MiR-128-3p inhibitor +si-control.

### Verification of the effects of MiR-128-3p *in vivo*

The rheumatoid arthritis mouse model was joint injection of MiR-128-3p inhibitor. The peripheral blood was used to detect the expression of TNFAIP3. The results revealed that the arthritis score was lower in MiR-128-3p inhibitor group than that in control (Figure 5A). The expression of MiR-128-3p was also decreased in MiR-128-3p inhibitor group (Figure 5B), while the expression of TNFAIP3 was increased in MiR-128-3p inhibitor group (Figure 5C). The results indicated that down-regulated MiR-128-3p protected joint against arthritis.

**Figure 5:** *In vivo* experiments to verify the expression of MiR-128-3p and TNFAIP3 Arthritis mice were injected with MiR-128-3p inhibitor. (**A**) The arthritis scores were determined every 3 days. (**B**) The expression of MiR-128-3p was determined using real-time PCR. (**C**) The TNFAIP3 was determined using Western blot; *P<0.05 vs. NC.

## Discussion

MiRNAs have been identified to mediate various process in body, the dysregulated miRNAs were often resulted in the diseases. For example, miR-486-5p served as a diagnostic marker in cervical cancer [26]; down-regulated miR-221-3p is associated with the poor prognosis of breast cancer [27]; miR-204-3p is a factor that induced familial mediterranean fever [28]; miR-146a and miR-155 showed dysregulated in oral lichen planus [29]. In addition, miRNA mediated inflammation in diseases, for example, miR-124 mediated the inflammatory pathogenesis of Parkinson’s disease [30]; miR-100 suppressed chronic vascular inflammation by stimulation of endothelial autophagy [31]. In addition, miR-548a-3p regulates the inflammatory response of RA by regulating the activity of TLR4/NF-κB signaling pathway [32]. MiR-10a-5p regulated joint inflammation in synoviocytes [33]. MiR-128-3p mediated the inflammation of rat kidney cells [19], and MiR-128-3p is a novel candidate oncogenic marker in T-cell acute lymphoblastic leukemia [34]. In the present study, MiR-128-3p was significantly increased in T cells of RA, indicating the potential role of MiR-128-3p in RA.

To further explore the potential role of MiR-128-3p on RA, the TNFAIP3 a negative regulator of NFκB activation was employed. TNFAIP3 was first discovered in human umbilical vein endothelial cells, and then researchers found that overexpressed TNFAIP3 dramatically suppressed the activation of NF-κB signaling pathway in various responses, such as the megakaryocytopoiesis [35], the differentiation of THP-1 cells [36], as well as the inflammation [37]. However, the potential targets between MiR-128-3p and TNFAIP3 were still did not documented. In the present study, we first found that TNFAIP3 was dominantly decreased in the T cells of RA. We further explored the potential role between MiR-128-3p and TNFAIP3. The online Targetscan predicted that MiR-128-3p bind with the TNFAIP 3′-UTR, the luciferase reporter assay further demonstrated that TNFAIP3 is a target gene of MiR-128-3p. The present study first identified the target relationship between TNFAIP3 and MiR-128-3p, indicating that MiR-128-3p mediated the mechanism of RA through regulating the expression of TNFAIP3.

The signaling pathway of NF-κB is widely participated in human body processes. Preliminary studies have identified that NF-κB is a key marker of RA in inflammation response [7,8]. Tumor necrosis factor-α (TNF-α) plays a critical role in TNFAIP3 suppressing the activity of NF-κB pathway [38]. The present study found that the knockdown of MiR-128-3p significantly decreased the p-IkBα, while due to that IkBα is a key marker in NF-κB pathway, thus we inferred that MiR-128-3p knockdown significantly decreased the activity of NF-κB pathway. Furthermore, knockdown of MiR-128-3p significantly promoted the expression of TNFAIP3, while cells co-transfected with MiR-128-3p inhibitor and si-TNFAIP3 altered the level of p-IkBα, indicating that MiR-128-3p regulated the NF-κB pathway is through regulating the expression of TNFAIP.

Inflammatory response is the main character of RA. From the present study, we found that the inflammatory cytokines IL-6 and IL-17 were significantly increased in T cells of RA, knockdown of MiR-128-3p significantly decreased the levels of IL-6 and IL-17, while cells co-transfected with MiR-128-3p inhibitor and si-TNFAIP3 abolished the effects of MiR-128-3p inhibitor, indicating that MiR-128-3p regulated the inflammatory response of RA is through regulating the expression of TNFAIP. The abnormally activity of T cells is also the main feature of RA [7]. The CD69 and CD25 is the main marker of T cells, thus, to examine the levels of CD69 and CD25 is important for measuring the activity of T cells. Here, we found that the knockdown of MiR-128-3p significantly decreased the ratio of CD69 and CD25, indicating that MiR-128-3p negatively regulated the activity of T cells.

In summary, the present study explored the potential mechanism of MiR-128-3p in RA, with the results of MiR-128-3p were significantly increased, the T cells and the NF-κB signaling pathway were activated, while down-regulating the expression of MiR-128-3p significantly suppressed the activation of T cells and the NF-κB signaling pathway, which was mediated by TNFAIP3, and further relieved the symptom of RA. The present study uncovered the mechanism of MiR-128-3p on RA, which provided great help for RA exploration. However, further study to verify the clinical use of MiR-128-3p for RA therapy is urgent.

## Abbreviations

CRP: C-reactive protein
DAS28: mean disease activity score in 28 joints
ELISA: enzyme-linked immunosorbent assay
ESR: erythrocyte sedimentation rate
IL: interleukin
PBMC: peripheral blood mononuclear cell
RA: rheumatoid arthritis
RF: rheumatoid factor
TNFAIP3: tumor necrosis factor-α-induced protein 3
